# Antioxidant Mechanism of Renal and Hepatic Failure Prevention Related to Paracetamol Overdose by the Aqueous Extract of *Amblygonocarpus andongensis* Stem Bark

**DOI:** 10.1155/2022/1846558

**Published:** 2022-07-21

**Authors:** O. Baponwa, A. P. Amang, C. Mezui, B. B. Koubala, G. T. Siwe, V. L. Vandi, P. V. Tan

**Affiliations:** ^1^Department of Biological Sciences, Faculty of Science, University of Maroua, P.O. Box 814, Maroua, Cameroon; ^2^Department of Biological Sciences, Higher Teachers' Training College, University of Yaoundé I, P.O. Box 047, Yaoundé, Cameroon; ^3^Department of Chemistry, Faculty of Science, University of Maroua, P.O. Box 814, Maroua, Cameroon; ^4^Department of Animal Biology and Physiology, Faculty of Science, University of Yaoundé I, P.O. Box 812, Yaoundé, Cameroon

## Abstract

Paracetamol is a commonly used analgesic/antipyretic whose long-term intake or overdose is associated with renal and hepatic injuries. The aim of this study was to determine the hepatonephroprotective mechanisms of the aqueous extract of *Amblygonocarpus andongensis* stem bark (AEAASB) on renal and hepatic failure resulting from paracetamol overdose. Forty-five rats were divided into nine groups (*n* = 5); these were treated once daily for 8 days with 5 ml/kg distilled water (normal, negative, and satellite controls); 0.9% normal saline and 140 mg/kg N-acetyl-cysteine (positive controls); 125, 250, and 500 mg/kg AEAASB (test groups); and 500 mg/kg AEAASB (satellite test). On day 8 after different treatments, hepatonephrotoxicity was induced in all the groups except the normal group by oral administration of a single dose of paracetamol (1000 mg/kg). Urinary, hematological, serum, and oxidative stress parameters and *in vitro* antioxidant activity of AEAASB were evaluated. Histological sections of the liver and kidney were performed. AEAASB significantly decreased urea, creatinine, transaminases, alkaline phosphatase, and bilirubin (*p* < 0.001) at 500 mg/kg compared to the negative control. Significant decreases in hepatic (*p* < 0.01) and renal (*p* < 0.001) malondialdehyde levels were associated with increases in superoxide dismutase, catalase, and reduced glutathione levels in 500 mg/kg AEAASB compared with the negative control. Histological analysis showed that AEAASB prevented paracetamol-induced renal and liver tissue damage. Furthermore, AEAASB revealed a very strong antioxidant activity (inhibitory concentration 50 = 180 *μ*g/ml, antioxidant activity index = 5.55) with an ability to scavenge 63.03% 2,2-diphenyl-2-picrylhy-drazyl radical and reduced ferric iron by 52.68 mgEqVitC/100 g DM. The hepatonephroprotective effect of AEAASB might result from its ability to improve the antioxidant status through the stimulation of antioxidant factors and the scavenging of free radicals. This property could be ascribed to the presence of some classes of bioactive compounds such as phenolic compounds in great amounts.

## 1. Introduction

Paracetamol, well known for its analgesic and antipyretic properties, is widely used in both clinical and self-medication contexts [1]. Prolonged use or overdose of paracetamol is associated with renal and hepatic damages [2, 3]. Hepatic damage due to the toxicity of this drug can progress to fulminant hepatic failure, which can lead to death [4]. Although nephrotoxicity in paracetamol overdose is less frequent than hepatotoxicity, renal damage can occur and sometimes be deadly [5].

At therapeutic dose, paracetamol is metabolized by glucuronidation and sulfation in the liver. These phase II reactions release water-soluble metabolites that are excreted by the kidneys [6]. Only a very small portion is eliminated unchanged in the urine. Residual paracetamol (approximately 5-9%) is oxidized by cytochrome P450 (CYP-450) enzymes, mostly CYP 2E1 to N-acetyl-p-benzoquinone imine (NAPQI) which is a highly reactive intermediate metabolite [3]. NAPQI is then reduced by glutathione and excreted by the kidneys as mercapturic acid, a relatively benign compound [7].

In the case of paracetamol overdose, sulfate and glutathione stores are depleted. A larger amount of the drug is then headed to the CYP-450 mixed-function oxidase system, generating more NAPQI [7]. Excessive production of this metabolite leads to increased toxicity, leaving large amounts of free reactive species. These electrophilic intermediates then form adducts with sulfhydryl and glutathione groups on cellular proteins [8]. The process disturbs homeostasis and leads to the activation of caspases and lysosomal enzymes, which trigger cell death by tissue necrosis [6].

The clinical management of paracetamol-induced hepatotoxicity consists of the administration of N-acetyl-cysteine (NAC) [4, 6, 9] which is metabolized to cysteine and increases the hepatic intracellular glutathione level [9]. Therefore, NAC has a clear role in the prevention and treatment of paracetamol-induced liver necrosis, but does not have protective effects against nephropathy [10]. According to recommendations of Kidney Disease Improving Global Outcomes (KDIGO) in 2012, regular saline intake can reduce the risks associated with drug-induced nephrotoxicity [11].

As the damage induced by paracetamol is mainly oxidative, natural compounds with antioxidant activity could be used as alternative treatments for paracetamol-induced hepatorenal toxicity [6]. Several studies have shown the efficacy of medicinal plant extracts on paracetamol-induced toxicity, including the works of Sudip et al. [12], Soliman et al. [13], and Al-Asmari et al. [14], which showed, respectively, the protective effects of *Citrus macroptera* fruit extracts, *Ocimum basilicum* leaves, and *Phoenix dactylifera* pollen on paracetamol-induced hepatorenal toxicity in rats.

*Amblygonocarpus andongensis* (Fabaceae) is a vascular plant from tropical regions of Africa widely used for its therapeutic virtues [15]. This plant has been classified among those with a powerful antioxidant activity [16]. Ethnomedicinal studies have revealed the use of *A*. *andongensis* bark in the treatment of ulcers, diarrhea, inflammation [17], diabetes, and hypertension [18]. Previous studies have shown analgesic [19], antipsychotic [20], and antidiarrheal properties of *A*. *andongensis* stem bark extract [21]. In Cameroon, information from traditional therapists suggests the use of this plant for the treatment of wounds, inflammation, jaundice, and kidney failure. The aim of this study was to elucidate the hepatonephroprotective mechanism of the aqueous extract of *A. andongensis* stem barks (AEAASB) on renal and hepatic failure resulting from an overdose of paracetamol.

## 2. Material and Methods

### 2.1. Plant Material

The stem barks of *A. andongensis* were collected in the locality of Gouna (Lagdo sub-Division, Benoue Division, North region, Cameroon) (08° 31′ 02.6″ N and 13° 33′ 44.3″ E). The samples were identified by Dr. Damolai Gounkagou Botanist at the Department of Biological Sciences of the Higher Teachers' Training College of the University of Yaoundé I and by Mrs. Ngwa Adeline Neh of the Herbarium of Garoua Wildlife School by comparing with existing specimens recorded under reference no. HEFG/1736. The collected barks were washed, weighed, shade-dried at room temperature, and then reduced into a fine powder. Five hundred grams (500 g) of this powder was dissolved in 3.5 liters of distilled water and boiled for 15 minutes. The decoction was allowed to cool for 45 minutes and then filtered through Whatman paper N°3. The obtained filtrate was evaporated using an oven at 50°C for 24 hours. A mass of 65.47 g of the extract was obtained representing a yield of 13.09%.

### 2.2. Animal Material

The experiment was carried out on male Wistar rats strains aged 12-14 weeks and with an average weight of 200 ± 20 g. These animals were raised at the Animal House of the Laboratory of Biological Sciences of the University of Maroua, Cameroon. They were housed in cages covered with wire mesh and maintained at room temperature with a natural light/dark cycle. They received a standard diet with unlimited access to tap water daily. Prior authorization for the use of laboratory animals in this study has obtained from Cameroon National Ethics Committee (Reg. N. FWA-IRB 00001954). The use, handling, and care of animals were done in adherence to the European convention for the protection of vertebrate animals used for experimental and other purposes [22].

### 2.3. Phytochemical Screening of AEAASB

The determination of the classes of compounds contained in AEAASB was carried out following the protocol described by Harborne [23]. The amounts of total phenolic compounds, total flavonoids, tannins, alkaloids, and terpenoids were estimated by the Folin-Ciocalteu [24], aluminum chloride (AlCl_3_) colorimetric [25], vanillin [26], methanol colorimetric [27], and chloroform colorimetric methods [28], respectively.

### 2.4. Evaluation of the In Vitro Antioxidant Activity of AEAASB

To determine the *in vitro* antioxidant activity of AEAASB, the 2,2-diphenyl-2-picrylhy-drazyl (DPPH) free radical scavenging activity [29] and the ferric reducing antioxidant power (FRAP) method [30] were evaluated. The inhibitory concentration 50 (IC_50_) was determined graphically using the DPPH method with the AEAASB concentration range of 0-200-400-600-800-1000 *μ*g/ml. In order to characterize the antioxidant activity of AEAASB, its antioxidant activity index (AAI) was evaluated according to the formula below and ranked according to the scale (poor activity < 0.5 < moderate < 1 < strong < 2 < very strong) of Scherer and Godoy [31].

(1) $$\begin{array}{c} \text{AAI}=\frac{\left[\text{DPPH}\right]}{{\text{IC}}_{50}}, \end{array}$$

(2) $$\begin{array}{c} \left[\text{DPPH}\right]=\text{final concentration of DPPH in the reaction},{\text{IC}}_{50}=\text{inhibitory concentration }50. \end{array}$$

### 2.5. Induction of Hepatorenal Toxicity

Forty-five (45) rats were divided into nine groups of five animals each. They received once daily *per os* for 8 days, 5 ml/kg of distilled water (normal, negative, and satellite controls), 5 ml/kg of 0.9% normal saline (positive control PS), 140 mg/kg of NAC (positive control NAC), AEAASB at 125, 250, and 500 mg/kg (test groups), and AEAASB 500 mg/kg (satellite test). On the 8^th^ day, one hour after the different treatments, a single dose of paracetamol (1000 mg/kg) was administered orally to all the animals except those of the normal control group (modified protocol of Canayakin et al. [6]). Immediately, all the animals except the satellite groups were fasted, and urine from each animal was collected for 24 hours using individual metabolic cages [32]. The animals were sacrificed under ketamine (2.5 mg/kg, *i.p*)/diazepam (5 mg/kg, *i.p*) anesthesia after 24 hours of fasting.

For the satellite groups of animals, urine collection and sacrifice were performed two weeks later following the same procedure.

### 2.6. Collection of Blood and Organ Samples

After rupture of the jugular vein, blood samples from each animal were collected in EDTA and dry tubes, for the analysis of hematological and biochemical parameters, respectively. Some organs (kidney, liver, heart, spleen, testes, lungs, and stomach) of each animal were removed and weighed to determine their relative weights [32, 33]. One kidney and part of the liver were used to prepare tissue homogenates [33]. The other kidney and the rest of the liver were gently rinsed in saline (0.9%) and conserved in 10% formaldehyde for histological analysis [34].

### 2.7. Urinary Analysis

Urinary parameters such as pH, osmolarity, and protein levels were measured using Urinalysis 11A Reagent Strips (ACON Laboratories Inc., USA). Urine flow rate (ml/min) was calculated according to the method of Bazzano et al. [35].

### 2.8. Analysis of Hematological and Serum Parameters

Total white blood cells, lymphocytes, granulocytes, red blood cells, hemoglobin, platelets, and mean corpuscular hemoglobin concentration of the animals were determined by blood count, using the Mindray BC-2800 hematology autoanalyzer. Serum biochemical parameters (creatinine, uremia, aspartate aminotransferase (ASAT), alanine aminotransferase (ALAT), alkaline phosphatase (ALP), and bilirubin) were measured using commercial kits (SGMitalia S.r.L, Italy). Glomerular filtration was assessed by creatinine clearance (Clcr) [35] according to the following formula:

(3) $$\begin{array}{c} \text{Clcr}\left(\text{ml}/\min\right)=\frac{\text{Urine creatinine }\left(\text{mg}/\text{dl}\right)\text{ x Urine flow rate }\left(\text{ml}/\min\right)}{\text{Serum creatinine }\left(\text{mg}/\text{dl}\right)}. \end{array}$$

### 2.9. Determination of Some Parameters of Oxidative Stress and Nitric Oxide (NO)

To carry out the assays of some parameters of oxidative stress, the kidney and liver homogenates were prepared by grinding 0.5 g of each organ in 2.8 ml of phosphate buffer solution (0.2 M, pH 7.4, pKa 7.2). Assays of total protein [36], NO [37], malondialdehyde (MDA) [38], superoxide dismutase (SOD) [39], catalase (CAT) [40], and reduced glutathione (GSH) [41] were performed from the kidney and liver homogenates.

### 2.10. Histopathological Examination

The histological sections of the liver and kidney were performed using the hematoxylin-eosin staining technique. The organs were cut and placed in cassettes and dehydrated. The tissues were solidified in moulds filled with molten paraffin. The sections of 5 *μ*m thickness were made with a microtome. After drying for 24 hours, the slides were stained by the hematoxylin-eosin. Note that hematoxylin (basophilic) stains the nuclear components blue-black and eosin (acidophilic) stains the cytoplasmic components pink-red. The stained sections were observed under a light microscope, and photographs were taken [42, 43].

### 2.11. Data Analysis

All the data were analysed by the one-way ANOVA test except for the relative evolution of weight which was analysed by the two-way ANOVA test followed by the Tukey posttest using GraphPad Prism software version 8.0.1. The results were expressed as mean ± standard error on mean, and the differences between the groups were significantly fixed at *p* < 0.05.

## 3. Results

### 3.1. Results of Phytochemical Screening of AEAASB

The qualitative phytochemical screening of AEAASB revealed the presence of phenolic compounds (flavonoids and tannins), terpenoids, and alkaloids. The quantification of classes of compounds showed that AEAASB contains mostly polyphenols (74.13 mgEqAG/100 g DM) (Table 1).

### 3.2. In Vitro Antioxidant Activity of AEAASB

The results of *in vitro* antioxidant activity showed that AEAASB (700 *μ*g/ml) scavenged 63.03% of DPPH• radical (Figure 1) and reduced ferric iron by 52.68 mgEqVitC/100 g DM. The IC_50_ of AEAASB following the DDPH method was 180 *μ*g/ml. The AAI being 5.55, AEAASB presents a very strong antioxidant activity.

### 3.3. Effect of AEAASB on the Body Weight Evolution

Figure 2 shows the evolution of the average body weights of the animals during the experiment. No significant difference (*p* > 0.05) was noted in the variation of body weights between the groups.

### 3.4. Effect of AEAASB on Food and Water Intake

Changes in food (Figure 3) and water intake (Figure 4) were not significantly different (*p* > 0.05) between the groups during the experiment.

### 3.5. Effect of AEAASB on the Relative Weight of Some Organs

Administration of paracetamol (1000 mg/kg) resulted in a significant increase (*p* < 0.05) of the liver relative weight in the negative control group compared to the normal control group (Figure 5). However, a significant decrease in the relative weight of this organ was noted in the group of the animals that received 500 mg/kg AEAASB (*p* < 0.05) and those of the satellite groups (*p* < 0.01) compared to the negative control.

### 3.6. Effect of AEAASB on Some Hematological Parameters

A significant increase in total leukocytes (*p* < 0.01) especially granulocytes (*p* < 0.001) associated with a significant decrease in red blood cells (*p* < 0.001), hematocrit (*p* < 0.001), and hemoglobin (*p* < 0.05) were noted in the negative control group compared to the normal control group (Table 2). However, treatment with AEAASB resulted in a significant decrease in total leukocytes (*p* < 0.05) and in granulocytes (*p* < 0.001) accompanied by a significant increase in red blood cells (*p* < 0.001), hematocrit (*p* < 0.001), and hemoglobin (*p* < 0.01) at the dose of 500 mg/kg compared to the negative control.

### 3.7. Effect of AEAASB on Some Parameters Related to Renal Function

The effect of AEAASB on the urinary parameters and some markers of renal function and renal creatinine clearance are presented in Table 3. The urine of the negative control group animals exhibited a significant decrease in creatinine level (*p* < 0.01) accompanied by an increase in protein level (*p* < 0.001) compared to the normal control group. However, in all animals treated with the different doses of the extract as well as in the satellite animals, a significant decrease in protein level was associated with an increase in urinary creatinine level (*p* < 0.001) compared to the negative control group was noted.

Paracetamol-induced nephrotoxicity resulted in a significant (*p* < 0.001) increase in serum creatinine, and urea levels were associated with a significant (*p* < 0.001) decrease in renal clearance in the negative control group compared to the normal control group (Table 3). However, treatment with AEAASB at doses of 250 and 500 mg/kg as well as in the satellite test group resulted in a significant decrease (*p* < 0.001) of creatinine and serum urea levels with an increase in renal clearance (*p* < 0.001) compared to the negative control.

### 3.8. Effect of AEAASB on Some Markers of Liver Function

Table 4 shows that the overdose administration of paracetamol (1000 mg/kg) resulted in a significant increase in ASAT, ALAT, ALP, direct, and total bilirubin levels (*p* < 0.001) in the negative control group compared to the normal control group. Contrariwise, AEAASB pretreatment significantly decreased the levels of these parameters in the 500 mg/kg AEAASB group as well as in satellite test group compared to the negative control (*p* < 0.001).

### 3.9. Effect of AEAASB on Some Parameters of Oxidative Stress, Total Protein, and NO Level in Renal and Hepatic Tissues

Table 5 shows the effect of AEAASB on some parameters of oxidative stress and NO level in renal and hepatic tissues. In the negative control group, paracetamol-induced nephrotoxicity was associated with a significant increase in MDA level (*p* < 0.001) accompanied by a significant decrease in SOD, CAT, and GSH levels (*p* < 0.01) as well as NO (*p* < 0.001) in the kidney compared to the normal control. However, administration of AEAASB at a dose of 500 mg/kg resulted in a significant decrease in MDA levels (*p* < 0.001) was associated with an increase in antioxidant levels (*p* < 0.001) as well as NO levels (*p* < 0.01) compared with the negative control.

After administration of paracetamol, there was a significant increase of hepatic MDA level (*p* < 0.01) was associated with a significant reduction in SOD (*p* < 0.01), CAT (*p* < 0.05), GSH (*p* < 0.001), and NO level (*p* < 0.001) in the negative control group compared to the normal control. However, pretreatment with AEAASB especially at the dose of 500 mg/kg resulted in a significant decrease in MDA level (*p* < 0.01) and an increase in SOD, CAT (*p* < 0.05), GSH (*p* < 0.001), and NO level (*p* < 0.01) in liver tissue compared to the negative control group (Table 5).

### 3.10. Effect of AEAASB on Renal Tissues of Rats

Histological sections of the kidneys of the animals in the normal control group showed normal structuring of the organ (Figure 6). In the negative control group, the administration of paracetamol resulted in renal alterations characterized by leukocyte infiltration, glomerular constriction, and dilatation of the urinary space. Glomerular constriction and dilatation of the urinary space were also noted in the test group receiving AEAASB 125 mg/kg. These alterations persisted in the satellite control rats. Only dilatation of the urinary space was noted in the rats of the positive control groups. However, these abnormalities were prevented in rats treated with AEAASB at 250 and 500 mg/kg and in the satellite test group.

### 3.11. Effect of AEAASB on Rat Liver Tissue

Histological analysis of the livers of the animals showed normal liver architecture in the normal control group (Figure 7). In the negative control group, leukocyte infiltration, dilatation, and congestion of portal vein were revealed. Dilatation and congestion of the portal vein were also noted in rats treated with AEAASB at 125 mg/kg. In the satellite control group, the portal vein dilatation persisted. However, these hepatic changes were prevented by AEAASB at 250 and 500 mg/kg and the reference products.

## 4. Discussion

Paracetamol or acetaminophen is a commonly used analgesic and antipyretic drug but is nephrotoxic at high doses [1, 8]. At therapeutic dose, approximately 85% of paracetamol undergo conjugation during phase II reactions in the liver to sulfate and glucuronide metabolites that are eliminated by the kidney [6, 44]. About 10% of paracetamol undergo phase I oxidation (mainly mediated by cytochrome 2E1) to NAPQI, which is normally conjugated with glutathione to mercapturic acid (nontoxic metabolites) [3, 7]. At high doses, paracetamol metabolism triggers potential mechanisms of toxicity [45]. The massive production of metabolites exacerbates toxicity by depleting glutathione and leaving large amounts of unbound reactive species. These electrophilic intermediates then form adducts with sulfhydryl and glutathione groups on cellular proteins [8]. This process leads to the activation of caspases and lysosomal enzymes that trigger liver cell death by necrosis, leakage of hepatocellular contents in the blood and liver failure [6, 10, 46].

The free radicals generated by NAPQI are the main actors of paracetamol toxicity and will stimulate lipid peroxidation [2] which leads to the release of numerous oxidation products such as MDA. Thus, the increase in MDA levels reflects tissue damage [47]. In addition to GSH depletion, NAPQI-induced oxidative stress can also lead to a reduction in the activity of certain antioxidant enzymes such as SOD and catalase [48, 49]. Hence, the high level of MDA and low levels of GSH, SOD, and CAT were observed in the group of untreated animals that received paracetamol (negative control). Substances that increase GSH, SOD, and CAT levels and decrease MDA levels are known to inhibit paracetamol-induced liver and kidney injury formation [13]. In the present study, AEAASB caused a significant decrease in MDA levels and an increase in SOD, CAT, and GSH levels in the liver and kidney. These results are in line with those obtained by Soliman et al. [13] who showed that the ethanolic extract of *O. basilicum* prevented paracetamol toxicity by enhancing the antioxidant status by decreasing MDA levels and increasing antioxidant enzyme levels in liver and kidney tissue. In addition, the results of *in vitro* antioxidant tests showed that AEAASB is a very strong antioxidant (IC_50_ = 180 *μ*g/ml, AAI = 5.55) that has the ability to scavenge 63.03% of DPPH• radicals and reduce ferric iron by 52.68 mgEqVitC/100 g DM. This important antioxidant capacity of the extract could be explained by its high polyphenol (74.13 mgEqAG/100 g DM) and alkaloid (51.27 mgEqQi/100 g DM) content. Indeed, alkaloids are powerful inhibitors of lipid peroxidation, and phenolic compounds are able to prevent oxidative stress by scavenging free radicals [50, 51]. This suggests that AEAASB could have inhibited lipid peroxidation, prevented depletion, and stimulated the production of antioxidant agents.

Paracetamol overdose also induces hepatotoxicity by the stimulation of hepatic lesions and inflammation characterized by an increase in liver weight and the level of liver function markers [52, 53]. Indeed, the rupture of the structural integrity of liver by cellular necrosis leads to the release of liver enzymes into the bloodstream [54]. At renal level, paracetamol overdose leads to an increase in serum creatinine and urea levels, indicating an alteration in renal function [55]. In addition, paracetamol-induced loss of functional integrity of renal cell membrane causes cellular leakage of proteins into the urine, leading to their appearance in large quantities in the urine. In animals treated with 500 mg/kg AEAASB and in the satellite test group, a significant decrease in relative liver weight of ASAT, ALAT, ALP, direct and total bilirubin, creatinine, serum urea, and urinary protein levels was associated with an increase of urinary creatinine, and renal clearance compared to the negative control group was noted. Results of the present study are similar to those of Al-Asmari et al. [14] who showed that *P. dactylifera* pollen prevented the loss of functional integrity of the liver and kidney cell membrane related to paracetamol toxicity in Wistar rats by decreasing the levels of liver and kidney function markers.

A significant increase in total leukocyte count, especially granulocytes, was associated with a significant decrease in red blood cell count, hematocrit, and hemoglobin was noted in the negative control group compared to the normal control. However, pretreatment with AEAASB (500 mg/kg) resulted in a significant decrease in leukocytes and a significant increase in red blood cells, hematocrit, and hemoglobin compared to the negative control as well as in the satellite group receiving this dose compared to the satellite control. Indeed, nephrotoxicity is related to an inflammatory aspect that causes an increase in the level of leukocytes in the blood which are recruited in the lesion site [56]. Furthermore, renal cells are secretors of erythropoietin, a stimulating hormone for the synthesis of red blood cells. The reduction of red blood cells number could be the result of compromised erythropoietin production as a result of the damage linked to paracetamol overdose [57]. According to Egbung et al. [56], the hematopoietic activity of *Vernonia calvoana* would be attributed to certain classes of compounds such as flavonoids, which could be the case with AEAASB.

Histopathological findings showed renal and hepatic alterations characterized by leukocytic infiltrations, glomerular constriction, dilatation of the urinary space, and dilatation and congestion of the hepatic portal vein (centrilobular necrosis) in the negative control group. The infiltrations result from the release of molecular signaling structures, including leukocytes, from the injured cells [58]. In addition, the glomerular constriction was associated with the dilatation of the urinary space would result from a decrease in glomerular filtration due to the constriction of the capillaries [59]. On the other hand, the centrilobular necrosis of the liver could be explained by the fact that the liver cells of the central zone are rich in CYP2E1 and, therefore, are the most sensitive to the lesions induced by paracetamol toxicity in overdose [4]. In the present study, the histopathological damage was the signs of renal and hepatic injury (24 hours after induction) originating from necrosis, which itself is not perceptible until several hours after cell death [60]. The animals treated with AEAASB at doses of 250 and 500 mg/kg and the satellite test group showed normal structural characteristics of the kidneys and liver. This is in agreement with the results of Dhibi et al. [61] and Allam et al. [62] who showed, respectively, that *Eucalyptus globulus* extract prevented renal alterations and alpha-lipoic acid prevented liver damage induced by paracetamol overdose administration in rats. These results suggest that AEAASB prevented paracetamol-induced damage.

## 5. Conclusion

Paracetamol overdose caused hepatic and renal damage resulting in increased levels of creatinine, urea, AST, ALT, ALP, direct and total bilirubin in blood, and protein in urine and decreased renal creatinine clearance in the negative control group compared to the normal control group. Paracetamol also caused an increase in MDA levels associated with a decrease in SOD, CAT, and GSH levels in the negative control group compared to the normal control group. A significant increase in leukocyte count associated with a decrease in red blood cell count, hematocrit, and hemoglobin was also noted in the negative control group compared to the normal control group. Treatment with AEAASB resulted in decreased MDA levels and increased SOD, CAT, and GSH levels compared to the negative control group. The extract also significantly decreased serum parameters and urinary protein levels and increased renal creatinine clearance compared to the negative control. AEAASB confers protection against paracetamol-induced hepatorenal toxicity by strengthening antioxidant status, *via* its ability to stimulate the production of antioxidant factors and scavenge free radicals. This property could be attributed to the presence of bioactive compounds, such as phenolic compounds, within this extract. However, due to the multifactorial etiology of hepatic and renal injury, our next investigations will evaluate the activity of this extract on other models of renal and hepatic injury and will associate the dosage of certain pro- and anti-inflammatory parameters. In addition, to reassure ourselves of the harmlessness of this extract for the population, the study of its toxicity will be carried out.

## Figures and Tables

**Figure 1:** *In vitro* antioxidant activity of AEAASB. (a) Percentage of DPPH• radical inhibition by AEAASB. (b) Capacity to reduce ferric iron by AEAASB (FRAP method). AEAASB: aqueous extract of *A. andongensis* stem bark; BHT: butylhydroxytoluene.

**Figure 2:** Effect of AEAASB on body weight. Positive control-PS: treated with 0.9% normal saline; positive control-NAC: treated with N-acetylcysteine; AEAASB 125, AEAASB 250, AEAASB 500: groups treated with aqueous extract of *A. andongensis* stem bark at doses of 125, 250, and 500 mg/kg, respectively; satellite AEAASB 500: treated with aqueous extract of *A. andongensis* stem bark at the dose of 500 mg/kg.

**Figure 3:** Effect of AEAASB on food intake. Positive control-PS: treated with 0.9% normal saline; positive control-NAC: treated with N-acetylcysteine; AEAASB 125, AEAASB 250, AEAASB 500: groups treated with aqueous extract of *A. andongensis* stem bark at doses of 125, 250, and 500 mg/kg, respectively; Satellite AEAASB 500: treated with aqueous extract of *A. andongensis* stem bark at the dose of 500 mg/kg.

**Figure 4:** Effect of AEAASB on water intake. Positive control-PS: treated with 0.9% normal saline; positive control-NAC: treated with N-acetylcysteine; AEAASB 125, AEAASB 250, AEAASB 500: groups treated with aqueous extract of *A. andongensis* stem bark at doses of 125, 250, and 500 mg/kg, respectively; satellite AEAASB 500: treated with aqueous extract of *A. andongensis* stem bark at the dose of 500 mg/kg.

**Figure 5:** Effect of AEAASB on the relative weight of some organs. Values are expressed as Mean ± SEM; positive control-PS: treated with 0.9% normal saline; positive control-NAC: treated with N-acetylcysteine; AEAASB 125, AEAASB 250, AEAASB 500: groups treated with aqueous extract of *A. andongensis* stem bark at doses of 125, 250, and 500 mg/kg, respectively; satellite AEAASB 500: treated with aqueous extract of *A. andongensis* stem bark at the dose of 500 mg/kg. ^♦^*p* < 0.05, significant difference compared to the normal control, ^∗^*p* < 0.05, ^∗∗^*p* < 0.01 significant difference compared to the negative control.

**Figure 6:** Microphotographs of rat kidneys (×200, hematoxylin-eosin stain). (a) Normal control. (b) Negative control. (c) Positive control treated with 0.9% normal saline. (d) Positive control treated with N-acetylcysteine. (e–g) Groups treated with aqueous extract of *A. andongensis* stem bark at doses of 125, 250, and 500 mg/kg, respectively. (h) Satellite control. (i) Satellite treated with aqueous extract of *A. andongensis* stem bark at the dose of 500 mg/kg. Gl: glomerulus; Us: urinary space; Dct: distal convoluted tubule; Pct: proximal convoluted tubule; LI: leukocyte infiltration; Gc: glomerular constriction; Dus: dilatation of the urinary space.

**Figure 7:** Microphotographs of rat livers (×200, hematoxylin-eosin stain). (a) Normal control. (b) Negative control. (c) Positive control treated with 0.9% normal saline. (d) Positive control treated with N-acetylcysteine. (e–g) Groups treated with aqueous extract of *A. andongensis* stem bark at doses of 125, 250, and 500 mg/kg, respectively. (h) Satellite control. (i) Satellite treated with aqueous extract of *A. andongensis* stem bark at the dose of 500 mg/kg. Hp: hepatic portal vein; He: hepatocyte; Ha: hepatic artery; Bd: bile duct; Sc: sinusoidal capillary; LI: leukocyte infiltration; DCh: dilatation and congestion of hepatic portal vein; Dh: dilatation of Hepatic portal vein.

**Table 1:** Results of the quantitative phytochemical screening of AEAASB.

Polyphenols (mgEqGA/100 g DM)	Flavonoids (mgEqQe/100 g DM)	Tannins (mgEqCa/100 g DM)	Alkaloids (mgEqQi/100 g DM)	Terpenoids (mgEqLu/100 g DM)
74.13 ± 0.71	61.27 ± 0.61	9.34 ± 0.59	51.27 ± 0.61	39.34 ± 0.58

mgEqAG: milligram equivalent of gallic acid; mgEqQe: milligram equivalent of quercetin; mgEqCa: milligram equivalent of catechin; mgEqQi: milligram equivalent of quinine; mgEqLu: milligram equivalent of lupeol; DM: dry matter.

**Table 2:** Effect of AEAASB on some hematological parameters.

	Total leukocytes (×10^9^/l)	Lymphocytes (%)	Granulocytes (%)	Red blood cells (×10^12^/l)	Hematocrit (%)	Hemoglobin (g/dl)	Blood platelets (×10^9^/l)
Normal control	0.78 ± 0.06	79.58 ± 1.02	7.48 ± 0.30	7.87 ± 1.23	41.44 ± 0.12	14.52 ± 0.51	430.60 ± 19.51
Negative control	1.14 ± 0.05^**♦♦**^	85.54 ± 0.36	11.42 ± 0.61^**♦♦♦**^	6.22 ± 1.78^♦♦♦^	29.34 ± 0.29^♦♦♦^	12.86 ± 0.23^♦^	483.20 ± 6.97
Positive control-PS	0.94 ± 0.05	80.94 ± 0.96	8.74 ± 0.32^∗∗^	7.31 ± 1.28^∗^	38.28 ± 0.12^∗∗∗^	13.54 ± 0.36	432.40 ± 9.63
Positive control-NAC	0.84 ± 0.07^∗^	88.84 ± 1.79	6.56 ± 0.62^∗∗∗^	7.26 ± 1.30^∗^	38.86 ± 0.00^∗∗∗^	14.12 ± 0.39	474.80 ± 15.72
AEAASB 125	1.08 ± 0.12	81.68 ± 1.67	11.02 ± 0.61	6.80 ± 1.00	36.42 ± 0.12^∗∗^	14.12 ± 0.46	480.60 ± 12.89
AEAASB 250	1.00 ± 0.04	80.40 ± 2.16	9.20 ± 0.46^∗∗^	7.11 ± 0.80^∗^	39.52 ± 0.27^∗∗∗^	14.28 ± 0.23	465.80 ± 15.73
AEAASB 500	0.80 ± 0.04^∗^	79.50 ± 0.54	8.20 ± 0.39^∗∗∗^	7.86 ± 1.06^∗∗∗^	40.30 ± 0.38^∗∗∗^	14.68 ± 0.25^∗∗^	421.80 ± 17.16
Satellite control	1.22 ± 0.04	81.76 ± 0.65	9.18 ± 0.43^∗^	6.86 ± 1.80	35.66 ± 0.30^∗∗^	14.70 ± 0.15^∗^	449.00 ± 21.70
Satellite AEAASB 500	0.90 ± 0.07**●**	79.76 ± 1.35	8.92 ± 0.44^∗∗^	7.58 ± 0.85^∗∗^	39.16 ± 0.31^∗∗∗^	14.68 ± 0.27^∗^	452.60 ± 15.34

Values are expressed as Mean ± SEM; positive control-PS: treated with 0.9% normal saline; positive control-NAC: treated with N-acetylcysteine; AEAASB 125, AEAASB 250, AEAASB 500: groups treated with aqueous extract of *A. andongensis* stem bark at doses of 125, 250, and 500 mg/kg, respectively; satellite AEAASB 500: treated with aqueous extract of *A. andongensis* stem bark at the dose of 500 mg/kg. ^♦^*p* < 0.05, ^♦♦^*p* < 0.01, ^♦♦♦^*p* < 0.001 significant difference compared to normal control, ^∗^*p* < 0.05, ^∗∗^*p* < 0.01, ^∗∗∗^*p* < 0.001 significant difference compared to negative control, ^●^*p* < 0.05 significant difference compared to satellite control.

**Table 3:** Effect of AEAASB on some parameters related to renal function.

	Urine output (ml/min ×10^−2^)	Urinary creatinine (mg/dl)	Urinary pH	Urinary osmolarity	Urinary protein (mg/dl)	Creatinine serum (mg/dl)	Urea serum (mg/dl)	Renal clearance (ml/min)
Normal control	0.80 ± 0.02	26.52 ± 1.36	6.30 ± 0.12	1.02 ± 0.00	100.0 ± 0.00	0.34 ± 0.03	53.71 ± 8.95	0.63 ± 0.03
Negative control	0.80 ± 0.01	19.58 ± 0.92^**♦♦**^	6.90 ± 0.29	1.02 ± 0.00	300.0 ± 0.00^**♦♦♦**^	2.51 ± 0.13^**♦♦♦**^	146.30 ± 8.11^**♦♦♦**^	0.06 ± 0.00^**♦♦♦**^
Positive control-PS	0.80 ± 0.01	29.54 ± 1.17^∗∗^	6.30 ± 0.12	1.03 ± 0.00	260.0 ± 40.00	1.60 ± 0.13^∗∗∗^	135.70 ± 10.96	0.15 ± 0.01^∗^
Positive control-NAC	0.76 ± 0.01	29.52 ± 2.55^∗∗^	6.00 ± 0.00	1.03 ± 0.00	100.0 ± 0.00^∗∗∗^	1.71 ± 0.17^∗∗∗^	134.30 ± 12.04	0.31 ± 0.02^∗∗∗^
AEAASB 125	0.77 ± 0.00	29.48 ± 0.59^∗∗∗^	6.70 ± 0.12	1.02 ± 0.00	140.0 ± 40.00^∗∗∗^	1.37 ± 0.08^∗∗∗^	78.31 ± 5.41^∗∗∗^	0.17 ± 0.01^∗^
AEAASB 250	0.77 ± 0.02	33.08 ± 2.67^∗∗∗^	6.50 ± 0.27	1.03 ± 0.00	100.0 ± 0.00^∗∗∗^	0.79 ± 0.13^∗∗∗^	70.85 ± 3.63^∗∗∗^	0.38 ± 0.02^∗∗∗^
AEAASB 500	0.87 ± 0.04	31.68 ± 1.72^∗∗∗^	6.50 ± 0.38	1.02 ± 0.00	100.0 ± 0.00^∗∗∗^	0.53 ± 0.05^∗∗∗^	67.14 ± 3.80^∗∗∗^	0.53 ± 0.03^∗∗∗^
Satellite control	0.84 ± 0.02	31.10 ± 0.32^∗∗∗^	6.70 ± 0.30	1.02 ± 0.00	180.0 ± 48.99^∗∗^	0.85 ± 0.10^∗∗∗^	152.60 ± 10.33	0.30 ± 0.03∗∗∗
Satellite AEAASB 500	0.81 ± 0.03	32.28 ± 1.68^∗∗∗^	7.00 ± 0.31	1.01 ± 0.00	100.0 ± 0.00^∗∗∗^	0.582 ± 0.04^∗∗∗^	78.34 ± 4.88^∗∗∗^^**●●●**^	0.45 ± 0.03^∗∗∗^^**●●**^

Values are expressed as Mean ± SEM; positive control-PS: treated with 0.9% normal saline; positive control-NAC: treated with N-acetylcysteine; AEAASB 125, AEAASB 250, AEAASB 500: groups treated with aqueous extract of *A. andongensis* stem bark at doses of 125, 250, and 500 mg/kg, respectively; Satellite AEAASB 500: treated with aqueous extract of *A. andongensis* stem bark at the dose of 500 mg/kg. ^♦♦^*p* < 0.01, ^♦♦♦^*p* < 0.001 significant difference compared to the normal control, ^∗^*p* < 0.05, ^∗∗^*p* < 0.01, ^∗∗∗^*p* < 0.001 significant difference compared to the negative control, ^●●^*p* < 0.01, ^●●●^*p* < 0.001 significant difference compared to the satellite control.

**Table 4:** Effect of AEAASB on some markers of liver function.

	ASAT (UI/ml)	ALAT (UI/ml)	Alkaline phosphatase (UI/ml)	Direct bilirubin (*μ*mol/l)	Total bilirubin (*μ*mol/l)
Normal control	135.60 ± 7.56	44.20 ± 2.03	110.80 ± 3.91	9.76 ± 0.28	13.68 ± 0.60
Negative control	209.60 ± 7.96^♦♦♦^	77.00 ± 2.95^**♦♦♦**^	172.30 ± 9.85^♦♦♦^	17.08 ± 0.44^♦♦♦^	21.10 ± 0.85^♦♦♦^
Positive control-PS	163.10 ± 12.74^∗∗^	72.60 ± 4.74	143.50 ± 8.07^∗^	16.36 ± 0.77	19.24 ± 1.29
Positive control-NAC	151.70 ± 9.98^∗∗∗^	54.80 ± 3.45^∗∗∗^	126.50 ± 9.35^∗∗∗^	11.26 ± 0.73^∗∗∗^	13.84 ± 0.37^∗∗∗^
AEAASB 125	161.00 ± 13.22^∗∗^	66.60 ± 3.58	153.50 ± 5.97	13.40 ± 0.26^∗∗∗^	20.36 ± 0.99
AEAASB 250	148.80 ± 14.22^∗∗∗^	54.80 ± 4.14^∗∗∗^	133.70 ± 6.72^∗∗^	12.12 ± 0.59^∗∗∗^	18.18 ± 0.73^∗^
AEAASB 500	138.70 ± 9.06^∗∗∗^	45.60 ± 1.57^∗∗∗^	112.40 ± 4.01^∗∗∗^	10.82 ± 0.46^∗∗∗^	13.84 ± 0.45^∗∗∗^
Satellite control	166.30 ± 3.15^∗∗^	70.60 ± 2.77	153.10 ± 4.20^∗∗∗^	12.66 ± 0.75^∗∗∗^	16.36 ± 0.56^∗∗∗^
Satellite AEAASB 500	143.80 ± 13.26^∗∗∗^	50.00 ± 2.77^∗∗∗^^**●●●**^	118.40 ± 5.18^∗∗∗^^●●^	9.96 ± 0.32^∗∗∗^^●●^	13.92 ± 0.57^∗∗∗^

Values are expressed as Mean ± SEM; positive control-PS: treated with 0.9% normal saline; positive control-NAC: treated with N-acetylcysteine; AEAASB 125, AEAASB 250, AEAASB 500: groups treated with aqueous extract of *A. andongensis* stem bark at doses of 125, 250, and 500 mg/kg, respectively; satellite AEAASB 500: treated with aqueous extract of *A. andongensis* stem bark at the dose of 500 mg/kg. ^♦♦♦^*p* < 0.001 significant difference compared to the normal control, ^∗^*p* < 0.05, ^∗∗^*p* < 0.01, ^∗∗∗^*p* < 0.001 significant difference compared to the negative control, ^●●^*p* < 0.01, ^●●●^*p* < 0.001 significant difference compared to the satellite control.

**Table 5:** Effect of AEAASB on some parameters of oxidative stress, total protein, and NO levels in kidney and liver tissues.

	Total protein	MDA (mmol/mg of protein)	SOD (U/mg of protein)	CAT (*μ*mol/min/mg of protein)	GSH (mmol/mg of protein)	NO (mmol/mg of protein)
Kidney tissue						
Normal control	23.35 ± 0.47	0.69 ± 0.03	19.98 ± 0.73	107.10 ± 2.96	2.14 ± 0.12	1.95 ± 0.06
Negative control	21.75 ± 0.90	0.99 ± 0.02^♦♦♦^	16.72 ± 0.44^♦♦^	88.75 ± 4.18^♦♦^	1.59 ± 0.03^♦♦^	1.42 ± 0.04^♦♦♦^
Positive control-PS	21.84 ± 0.46	0.83 ± 0.04^∗^	17.84 ± 0.93	101.50 ± 2.61	1.95 ± 0.16	1.62 ± 0.02
Positive control-NAC	20.80 ± 0.35	0.74 ± 0.04^∗∗∗^	19.23 ± 0.30^∗^	107.20 ± 3.39^∗^	2.40 ± 0.12^∗∗^	1.57 ± 0.03
AEAASB 125	21.44 ± 0.83	0.78 ± 0.05^∗∗^	17.83 ± 0.49	95.15 ± 3.67	2.63 ± 0.14^∗∗∗^	1.46 ± 0.07
AEAASB 250	21.42 ± 1.08	0.73 ± 0.03^∗∗∗^	18.97 ± 0.46^∗^	108.90 ± 4.62^∗∗^	2.93 ± 0.17^∗∗∗^	1.61 ± 0.04
AEAASB 500	22.51 ± 0.77	0.71 ± 0.04^∗∗∗^	20.72 ± 0.33^∗∗∗^	117.90 ± 4.27^∗∗∗^	3.45 ± 0.08^∗∗∗^	1.81 ± 0.08^∗∗^
Satellite control	22.43 ± 0.61	0.93 ± 0.05	16.79 ± 0.40	98.45 ± 2.98	1.81 ± 0.10	1.41 ± 0.05
Satellite AEAASB 500	22.45 ± 1.04	0.78 ± 0.03^∗∗^^●^	19.08 ± 0.51^∗^^●^	101.40 ± 2.32	2.36 ± 0.16^∗∗^^●^	1.58 ± 0.12
Liver tissue						
Normal control	19.48 ± 0.47	0.86 ± 0.02	21.88 ± 0.47	99.29 ± 6.90	3.19 ± 0.13	1.94 ± 0.06
Negative control	19.58 ± 0.59	1.23 ± 0.06^♦♦^	18.96 ± 0.66^♦♦^	75.21 ± 5.73^♦^	1.97 ± 0.13^♦♦♦^	1.28 ± 0.07^♦♦♦^
Positive control-PS	20.47 ± 0.40	1.16 ± 0.04	19.40 ± 0.46	83.03 ± 4.23	1.27 ± 0.27^∗^	1.53 ± 0.12
Positive control-NAC	20.35 ± 0.64	1.13 ± 0.07	19.41 ± 0.58	87.69 ± 6.76	2.58 ± 0.17^∗^	1.88 ± 0.06
AEAASB 125	18.78 ± 0.45	1.06 ± 0.06	19.40 ± 0.42	90.48 ± 5.09	1.93 ± 0.12	1.38 ± 0.02
AEAASB 250	20.36 ± 0.71	0.98 ± 0.06^∗^	20.84 ± 0.36	100.7 ± 0.91^∗∗^	2.42 ± 0.14	1.46 ± 0.05
AEAASB 500	20.83 ± 0.37	0.88 ± 0.05^∗∗^	22.08 ± 0.50^∗∗^	102.5 ± 3.68^∗∗^	3.48 ± 0.14^∗∗∗^	1.70 ± 0.05^∗∗^
Satellite control	19.89 ± 0.46	0.97 ± 0.06^∗^	21.02 ± 0.46	48.14 ± 3.08^∗∗∗^	1.15 ± 0.11^∗∗^	1.37 ± 0.04
Satellite AEAASB 500	18.97 ± 0.40	0.84 ± 0.07^∗∗∗^	21.46 ± 0.39^∗^	98.06 ± 2.76^∗^^●●●^	2.36 ± 0.23^∗∗∗^^●●●^	1.46 ± 0.09

Values are expressed as Mean ± SEM; positive control-PS: treated with 0.9% normal saline; positive control-NAC: treated with N-acetylcysteine; AEAASB 125, AEAASB 250, AEAASB 500: groups treated with aqueous extract of *A. andongensis* stem bark at doses of 125, 250, and 500 mg/kg, respectively; satellite AEAASB 500: treated with aqueous extract of *A. andongensis* stem bark at the dose of 500 mg/kg. ^♦^*p* < 0.05, ^♦♦^*p* < 0.01, ^♦♦♦^*p* < 0.001 significant difference compared to the normal control, ^∗^*p* < 0.05, ^∗∗^*p* < 0.01, ^∗∗∗^*p* < 0.001 significant difference compared to the negative control, ^●^*p* < 0.05, ^●●●^*p* < 0.001 significant difference compared to the satellite control.

## Data Availability

The data used to support the findings of this study are available from the corresponding author upon request.
